The article "Comparison of Hepatectomy and Hemangiomas Stripping on Patients with Giant Hepatic Hemangiomas" was retracted in 2023. Reasons: signs of a paper mill; compromised peer review; unreliable results or conclusions.

# Comparison of Hepatectomy and Hemangiomas Stripping on Patients with Giant Hepatic Hemangiomas

**DOI:** 10.1155/2022/1350826

**Published:** 2022-08-31

**Authors:** Zhiqi Yang, Chunyan Zhang, Zhiwen Li, Lang Wu, Minghao Li

**Affiliations:** ^1^Ningxia Medical University, Yinchuan 750004, Ningxia, China; ^2^Hepatobiliary Surgery of Ningxia Hui Autonomous Region People's Hospital, Yinchuan 750021, Ningxia, China

## Abstract

**Objective:**

To compare the value of a hepatectomy and hemangioma stripping on patients with giant hepatic hemangiomas.

**Methods:**

Seventy-four patients with giant hepatic hemangiomas were retrospectively analyzed from data collected from their hepatobiliary surgeries performed from June 2010 to June 2015 at the People's Hospital of Ningxia and the general hospital affiliated with Ningxia Medical University. The patients were divided into a hepatectomy group (37 patients) and a hemangioma-stripping group (37 patients). Conditions of each group were compared before and after surgery and comprised of surgery duration, intraoperative blood loss, blood transfusion, duration of hepatic blood occlusion, and hospital stay. Any complications after surgery, such as pleural effusions, bile leakage, and abdominal hemorrhage, were also observed.

**Results:**

In the hemangioma-stripping group, the surgery time was 2.38 ± 0.93 h, intraoperative blood loss was 889.19 ± 756.37, blood transfusion amount was 723.78 ± 801.14, the duration of hepatic blood occlusion 26.84 ± 17.30 min, and hospital stay was 16.19 ± 5.01 d. In the hepatectomy group, surgery time was 3.26 ± 1.16 h, intraoperative blood loss was 1551.35 ± 1755.88 mL blood transfusion amount was 1693.24 ± 2117.72 mL, duration of hepatic blood occlusion was 26.84 ± 17.30 min, and hospital stay was 16.19 ± 5.01 d. The difference between the groups was statistically significant (*P* < 0.05). The pleural effusion incident rate in the former group was lower than that of the latter group, and the difference was statistically significant.

**Conclusions:**

Hemangiomas stripping is an effective method by which to cure hepatic hemangioma, with the advantages being a relatively easy surgery with less patient trauma, rapid recovery, and fewer complications. This method should be used more often in clinical settings.

## 1. Introduction

Hepatic hemangioma is the most common benign tumor of the liver, with an incidence rate of 3–20% and a demonstration rate in autopsy of 0.4–7.4%14 [1, 2]. However, the exact pathologic mechanism by which hepatic hemangiomas appear is unclear. These vessel growths can appear at any age and are more common in middle-aged women.

The morbidity rate of men to women is 1 : 5 to 6. A hepatic hemangioma is a type of vascular malformation and is classified into cavernous hemangioma, sclerosing hemangioma, angioendothelioma, and capillary hemangioma according to the number of fibrous tissues [3]. Clinical cavernous hemangiomas, usually called hepatic hemangiomas, are the most common and are induced by liver sinusoids in the embryonic stages. Tumors can be of different sizes and can be single (most common) or multiple. In China, the tumor is graded according to the following three criteria: small cavernous hemangioma with a diameter <5.0 cm, large cavernous hemangioma.

Until now, there has been no one effective method by which hepatic hemangiomas are treated [4]. Surgery remains the main treatment method; however, how to assess the indications for surgery and select a safe and effective treatment method are the main concerns in clinics.

There are several surgical treatments for hemangioma, such as liver resection, hemangioma binding, hepatic artery ligation, radio frequency ablation, and liver transplantation. Of these, liver resection is the first choice of treatment.

There is major debate over the indications for hepatic hemangioma surgery and other therapeutic options. The most common and thorough way by which to cure the condition is to resect the hemangioma, which includes hepatectomy and hemangioma stripping [1]. However, with giant hepatic hemangiomas, surgery is dangerous and difficult. During surgery, the size, location, number of tumors, and relationship between the tumors and the adjacent tissues must be considered, especially for giant hepatic hemangiomas that are situated in the hilar area, because of the possibility of a massive hemorrhage during the surgery, which could endanger the patient's life. The key to a successful surgery is to choose a reasonable method and control any intraoperative blood loss. After the resection of a giant hepatic hemangioma, the complications are mainly abdominal hemorrhage, bile leakage, pleural effusions, and ascites. This study retrospectively analyzed the clinical data on 74 patients with giant hepatic hemangiomas who had hepatobiliary surgery from June 2010 to June 2015 at the Ningxia People's Hospital and the general hospital affiliated with Ningxia Medical University. Two surgical methods hepatectomy and hemangioma stripping are compared and discussed.

By comparing the two types of surgical treatment for giant hepatic hemangioma, clinical evidence for curing giant hepatic hemangiomas and guidance for choosing a reasonable and safe surgical method to reduce complications are provided.

## 2. Materials and Methods

### 2.1. General Information

The diagnostic criteria for being selected for the study were as follows:

1. Diameter of hepatic hemangioma≥10 cm and
2. Patient's pathologic examination and diagnosis after surgery of cavernous liver hemangioma.

Inclusion criteria:

1. The clinical findings were consistent with the diagnostic criteria of giant hemangioma of the liver;
2. There were obvious abdominal mass, anorexia, nausea, and vomiting and other symptoms;
3. Patients diagnosed by abdominal B-ultrasound, CT, MRI, liver histopathology, hepatic arteriography, patients with huge hepatic hemangioma;
4. There are indications for surgical treatment;
5. Written informed consent was obtained from all patients and agreed to participate in the study.

Exclusion criteria:

1. Patients with important organ failure;
2. Patients with definite contraindications;
3. Serious communication barriers;
4. Declined to participate in this study.

There were 17 male patients and 57 female patients between 26 and 69 years of age with a median age of 45 years. Before surgery, the liver function Child–Pugh score was “A”. The diameter of the tumors ranged from 10.0 to 24.9 cm, with an average of 12.5 cm.

Patients were divided into two groups as follows: hepatectomy (*n* = 37) and hemangioma stripping (*n* = 37). The hepatectomy group) comprised 10 males and 27 females, ages 31–63 years with a median age of 45 years. The tumor diameter of the hepatectomy group was between 10.0 and 18.1 cm, with an average size of 12.9 cm. The 37 patients in the hemangioma stripping group were comprised of 7 males and 30 females, ages 26–69 years, with a median age of 43 years. The tumor diameter of those in this group was from 10.0 to 24.9 cm, with an average of 12.1 cm.

Both groups had single and multiple tumors. The hepatectomy group had 16 cases of single tumor and 21 cases of multiple tumors; the hemangioma stripping group had 23 cases of single tumors and 14 cases of multiple tumors. There were 16 cases of cholecystectomy in the hepatectomy group and 10 cases in the hemangioma-tumor stripping group. One patient in each group had received a cholecystectomy prior to hemangioma surgery. In the hepatectomy group, there were 22 patients whose tumors were located in the left lobe, 12 whose tumors were located in the right lobe, and 3 whose tumors were throughout the entire liver. In the hemangioma stripping group, there were 9 patients whose tumors were located in the left lobe, 21 whose tumors were located in the right lobe, and 7 whose tumors were located throughout the entire liver. There was no significant difference in sex, age, and complicated hepatitis between the two groups (Table 1). The difference in the quantity and tumor diameter between the two groups was also not significant; however, there was a significant difference between the groups in the location of the tumor (*P* < 0.05) with more cases of left-lobe hepatectomy in the former group than in the latter group (Table 2 and 3).

### 2.2. Treatment Methods

#### 2.2.1. Hepatectomy

After general anesthesia and a subcostal incision, the falciform ligament, left and right triangular ligaments, coronary ligament, and round ligament were completely freed to fully expose the tumor and begin the hepatectomy regularly or irregularly.

#### 2.2.2. Hemangioma Stripping

After general anesthesia and a subcostal incision to fully expose the tumor, the round ligament, falciform ligament, left and right triangular ligaments, and coronary ligament were clamped, cut, and ligated. After the anatomy of the first hepatis porta and the second hepatis porta, indwell the band-blockade.

When stripping the tumor within 1.0 cm of normal liver tissue at the edge of the hepatic hemangioma, the liver capsule was cut first, and a tool holder was used to do a blunt separation along the gap between the tumor and normal liver tissue to the surface of the tumor. The vascular vessels and bile duct were clamped, cut, and ligated to reduce blood loss and create a biliary fistula. After having completely stripped the entire hemangioma, any bleeding was stopped and the wound was sutured.

### 2.3. Observation Indices

Presurgery observation indices comprised general conditions such as sex, age, presence of hepatitis, and the liver function before surgery.

The Child–Pugh system of classification was used to quantify liver reserve function. The status of the other indices serum bilirubin, plasma albumin, prothrombin prolong time, ascites, and hepatic encephalopathy were classified using three levels (1, 2, and 3). The five index scores were summed; the minimum score was 5 and the maximum was 15. According to the total score, the liver function was graded using an A, B, or C, which represented three types of liver damage by degree (the higher the score, the worse the liver reserve function). Conclusions were drawn from patient records and the results of laboratory tests.

The quantity, diameter, and location of the tumors were observed using abdominal ultrasonography, computed tomography (CT), and abdominal magnetic resonance imaging (MRI) results. The surgery duration, blood loss, blood transfusion amount, duration of hepatic blood occlusion, duration of hospital stay, and any additional cholecystectomies were taken from patient surgery reports. After surgery, any complications in the patients of both groups were noted, including pleural effusions, bile leakage, abdominal hemorrhage, and wound infection. All information was taken from the medical record, laboratory test results after surgery, and imaging reports.

### 2.4. Statistical Analyses

The data were analyzed using SPSS 17.0 (SPSS Inc., Chicago, IL, USA), The two independent samples measurement data measured by *x* ± *s* and enumeration data measured by rate are compared using Student's *t*-test and *X*^2^ test. (*P* < 0.05 indicated significance).

## 3. Results

### 3.1. Intraoperative Conditions

Surgery duration, blood loss and amount of blood transfused during surgery, duration of hepatic blood occlusion, and duration of hospital stay were obviously less in the hemangioma-stripping group than in the hepatectomy group, and the difference was significant (*P* < 0.05) (Table 4). In the hepatectomy group, there were 7 cases of unblocked hepatic blood and 30 of hepatic blood occlusion. Among 3 cases of selective semihepatic blood occlusion, the first hepatis porta occlusion (Pringle procedure) was performed on 27 patients. Of the hemangioma-stripping group, there were 2 cases of unblocked hepatic blood and 35 cases of hepatic blood occlusion. Amongst 2 cases of selective semihepatic blood occlusion, a first hepatis porta occlusion (Pringle procedure) was performed on 33 patients.

### 3.2. Postsurgery Conditions

Surgery on all patients was successful; however, there was one death after a hepatectomy during the perioperative stage, 10 cases of postsurgery pleural effusion, and 1 case of bile leakage; there was no abdominal hemorrhaging; In the hemangioma-stripping group, there were three cases of pleural effusion, two of bile leakage, and one of abdominal hemorrhaging. There were no deaths.

There was no significant difference in bile leakage, abdominal hemorrhage, and death of the patients between the two groups (*P* > 0.05). The incidence of pleural effusion in the hemangioma-stripping group was less than that in the hepatectomy group (*P* < 0.05) (Table 5).

### 3.3. Postsurgery Follow-Up

There was one death after hepatectomy during the perioperative stage, one case of hepatic hemangioma recurrence, 11 cases of no postsurgery follow-up, and 24 cases of full recovery. There was one death after the hemangioma-stripping surgery during the perioperative stage, one case of hepatic hemangioma recurrence, 9 cases of no postsurgery follow-up, and 26 cases of full recovery.

## 4. Discussion

The exact cause of hepatic hemangioma is still unknown, but congenital developmental abnormality is the most accepted theory [3, 5]. However, some scholars believe that because of an infection in the liver, the capillaries transform, leading to them becoming vacuolated, and peripheral vascular congestion, dilation, and stranding of regional blood circulation result in the cavernous expansion of the blood vessels. Some scholars find that all liver hemangiomas are derived from the hepatic artery system. Others observed that the estrogens involved with female puberty, pregnancy, oral contraceptives, and other circumstances could stimulate the growth of hemangiomas.

The progress of a hemangioma is usually slow and not of major concern. There are no symptoms when the tumors are small; however, they are often found during physical examinations and celiotomies. When the diameter of the hemangioma is > 5.0 cm, some patients might exhibit nonspecific symptoms in the abdomen, such as abdominal distension, stomachache, anorexia, or nausea, which are caused by hepatomegaly or compression of the stomach and intestine. Occasionally, the tumor ruptures and the pedicle reverses may result in acute abdominal pain. Spontaneous rupture and bleeding are very rare in large hemangiomas and seldom reported. Kasabach–Merritt syndrome, also known as “hemangioma with thrombocytopenia,” leads to decreased platelet counts and sometimes other bleeding problems. Biliary tract bleeding is rare but is also seen. Upper abdominal masses connected to the liver are a common feature of it, and are characterized as follows:

1. Smooth, moderate, or soft and lobulated;
2. Moving up and down freely with breathing;
3. A feeling of a capsule and compression of different degrees; and
4. Usually no or only mild tenderness. Sometimes a vascular murmur in the liver can be heard. Because of the lack of characteristic clinical manifestations of a hepatic hemangioma and lack of specificity in laboratory tests, a clinical diagnosis depends on CT scans, MRI scans, or other imaging examinations.

Recently, image diagnostic techniques have been highly developed, which has increased the diagnosis of hepatic hemangioma. B-mode ultrasound, CT, MRI, hepatic angiography, and radionuclide hepatic blood pool scanning can provide an exact diagnosis. A B-mode ultrasound is the most common method used, with an accuracy rate of 70–80%. Because this method is convenient, fast, and economical, it is often used for postsurgery follow-up [1]. However, the most accurate method is MRI, because it is 95% sensitive and nearly 100% accurate and provides a better method by which to confirm the disease. A liver biopsy is done only in cases that are difficult to diagnose by routine examination.

There is a major debate on the indications for hepatic hemangioma surgery and the therapeutic method, the most common and thorough of which is resection of the tumor [6, 7] including hepatectomy and hemangioma stripping [8]. Based on a report by Iacobas I, [9] the surgical indications of hepatic hemangiomas are as follows [10]:

1. Care should be taken when the patients are >50 years old, and no special treatment should be given to patients who have no obvious symptoms and no reduction in their quality of life. For patients >50 years old whose tumor is obviously enlarged, surgery can be considered.
2. It is difficult to differentiate a newly discovered hepatic hemangioma from other liver diseases. When faced with patients for whom there is no exact diagnosis of hepatic hemangioma, have tested positive for hepatitis, or who have a history of chronic liver disease, surgery should be considered.
3. If the diameter of the tumor is > 10 cm, appears with central necrosis, and has a risk of spontaneous rupture and bleeding, surgery should be considered; however, these situations are rare and cannot always be an indication of hepatic hemangioma.
4. If there are complications, such as stomachache, compression of adjacent organs, and Kasabach–Merritt syndrome, the tumor must be removed.
5. During pregnancy, the size of a hepatic hemangioma might increase and could rupture during delivery; therefore, the tumor should be removed, especially in young females.
6. For those who participate in sports such as boxing and soccer and those who might experience liver trauma, surgery should be considered to remove the tumor.
7. If patients suffer from intrahepatic multiple hemangiomas, resulting in hepatic dysfunction and Kasabach–Merritt syndrome with obvious bleeding, liver transplantation might be considered.

When the hepatic sinusoid is congested, its volume enlarges with expansive growth, which results in the formation of hemangiomas. Normal hepatocytes surrounding the tumor gradually shrink, leaving no normal hepatocytes visible in a pathological examination. There is a thin fibrous capsule between the tumor and normal hepatocyte, a clear boundary with surrounded by hepatic tissue. If the hepatic hemangiomas are cut between the outside of the fibrous capsule and normal liver tissue, they can be completely removed without damaging the normal liver tissues [11]. This is the foundation of the hemangioma-stripping procedure.

There are many advantages to this method as follows:

1. Because of the abundant blood supply of hepatic hemangiomas, hemorrhage during surgery is reduced, reducing the corresponding amount of intraoperative blood transfusion. When this method is used, patients with giant hepatic hemangiomas (>10 cm in diameter) can keep more normal liver tissue, the complication rate is low, and liver function recovers rapidly. There is a fibrous membrane between the hepatic hemangioma and tumor. If the tumor is cut along with the liver hemangioma capsule, the damage to the intrahepatic bile duct and blood vessels will be reduced, and bile leakage and the recurrence rate of intra-abdominal hemorrhage after surgery will be lower.
2. Tumors are completely stripped and the possibility of recurrence is reduced.
3. The surgery is simple, fast, and economical, and postsurgery recovery is rapid.

The complication rate is 13.1%. Large hemangiomas of the liver (diameter >10 cm) are usually close to the hepatic artery, portal vein, hepatic vein, postcava, aortaventralis, and biliary system and can spread to the first, second, and third hepatic portal. Slight carelessness could lead to massive hemorrhage and endanger a patient's life; therefore, adequate presurgery assessment and a reasonable procedure are the keys to a successful surgery. These are as follows:

1. Presurgery imaging: abdominal CT enhanced scanning can reveal the quantity, size, and location of the tumors and the relationships to adjacent blood vessels, the biliary tract, and other viscera. With the help of CT vascular remodeling, the relationship with surrounding blood vessels can be clearly defined. Based on the CT examination, which can diagnose 90% of cases, the surgical protocol can be prepared. If the bulb of NMR is also found, the diagnostic accuracy can be improved. [12].
2. Presurgery preparation: this should include liver function Child–Pugh classification, routine blood tests, and coagulation function. Patients who take aspirin ensure medication compliance. A red cell suspension and plasma must be prepared in advance in case of massive hemorrhage during surgery. [13].
3. Choice of methods: A hepatic hemangioma is a benign tumor having an abundant blood supply, and giant hepatic hemangiomas (diameter ≥10 cm), especially those located in the first, second, and third hepatic portal are at risk of the tearing the inferior vena cava and aorta abdominalis. Generally, a band is preset for portal trad clamping to protect from massive hemorrhage, so that the blood flowing into the liver can be quickly blocked to control bleeding. [14].

## 5. Conclusion

Among the 74 patients in this study, 9 had unblocked hepatic blood, 65 had hepatic blood occlusion, and 5 had selective hemihepatic blood flow occlusion; 60 cases had a block of the first hepatic portal. Hemihepatic blood flow occlusion blocks the blood on the lesion side from flowing into the liver and protects the normal liver from ischemia-reperfusion injury. During surgery, relatively stable hemodynamic changes and less visceral congestion provide enough time for surgeons to carefully process the section, which lays a good foundation for recovery. The method of occlusion is chosen according to the location, size, and degree of invasion of the tumors. Because a hepatic hemangioma is a type of benign tumor, intraoperative autotransfusion can be used.

Giant hepatic hemangiomas have an abundant blood supply, so surgical bleeding and its reduction must be considered. It is important to choose a suitable subcostal incision to provide an adequate view of the surgery area to carefully dissect the hilar structure. Hepatic portal blood occlusion provides a fast and effective way by which to control bleeding. During hemangioma stripping the boundary between the tumor and normal liver tissues must be delineated. The vascular and biliary tracts must be clamped, cut, and ligated. Care must be taken to avoid cutting the tumor or the normal liver tissue.

The data on this study indicate that hemangioma stripping is superior to hepatectomy in surgery duration, bleeding, and blood transfusion during surgery duration of hepatic blood occlusion, and duration of hospital stay. This method protects the normal liver so that patients recover faster with fewer complications. Except for patients with traumatic tumor hemorrhage and spontaneous tumor hemorrhage, extracellular membrane stripping can be used. Stripping of giant hemangiomas is safe, convenient, and cost-effective, and should be considered in clinical applications.

## Figures and Tables

**Table 1:** Comparison of the general conditions.

Groups	Total number	Sex (M/F)	Age	Hepatitis (Y/N)
Hepatectomy	37	10/27	46.86 ± 8.54	1/36
Hemangioma-stripping group	37	7/30	45.73 ± 9.74	1/36
*t*/*χ*^2^		0.687	0.533	0.000
*P*		>0.05	>0.05	>0.05

**Table 2:** Comparison of the tumors in patients.

Groups	Total number	Tumor (single/multiple)	Diameter (cm)	Location (left lobe/right lobe/entire liver)
Hepatectomy	37	16/21	12.882.83	22/12/3
Hemangioma-stripping	37	23/14	12.14 ± 3.09	9/21/7
*t*/*χ*^2^		2.656	1.078	9.506
P		>0.05	>0.05	<0.05

**Table 3:** Comparison of the tumor location in patients.

Group	Hepatectomy group	Hemangioma stripping group	*χ* ^2^	*P*
Left lobe	22	9	7.686	0.006
Right lobe	12	21		

Left lobe	22	9	5.333	0.021
Whole liver	3	7		

Right lobe	12	21	0.137	0.711
Whole liver	3	7		

**Table 4:** Comparison of the patient conditions and hospital stay.

Group	Number of patients	Surgery duration (h)	Intraoperative blood loss (mL)	Intraoperative blood transfusion (mL)	Hepative blood occlusion time (min)	Hospital stay (d)
Hepatectomy group	37	3.26 ± 1.16	1551.35 ± 1755.88	1693.24 ± 2117.72	26.84 ± 17.30	16.19 ± 5.01
Hemangioma stripping	37	2.38 ± 0.93	889.19 ± 756.37	723.78 ± 801.14	22.48 ± 10.87	14.84 ± 3.24
*t*/*F*		3.635	11.013	6.472	9.794	3.995
*P*		<0.05	<0.05	<0.05	<0.05	<0.05

**Table 5:** Patient complications after surgery.

Group	Number of cases	Pleural effusion (Y/N)	Bile leakage (Y/N)	Abdominal hemorrhage (Y/N)	Death (Y/N)
Hepatectomy	37	10/27	1/36	0/37	1/36
Hemangioma stripping	37	3/34	2/35	1/36	0/37
*χ* ^2^		4.573	0.347	1.014	1.014
*P*		<0.05	>0.05	>0.05	>0.05

## Data Availability

The data that support the findings of this study are available from the corresponding author upon reasonable request.

## References

[1] Oldhafer K. J., Habbel V., Horling K., Makridis G., Wagner K. C. (2020). Benign liver tumors. *Visual Medicine*.

[2] Toro A., Mahfouz A. E., Ardiri A. (2014). What is changing in indications and treatment of hepatic hemangiomas. A review. *Annals of Hepatology*.

[3] Zamparelli M. S., Rimola J., Montironi C. (2020). Hepatic epithelioid hemangioendothelioma: an international multicenter study. *Digestive and Liver Disease*.

[4] Jien H., Xiaohua L. (2021). Laparoscopic versus open surgery in the treatment of hepatic hemangioma: a meta-analysis. *Medicine (Baltimore)*.

[5] Keim D. W., Vokuhl C., Walz C. (2019). Activation of hedgehog signaling in aggressive hepatic hemangioma in newborns and infants. *Anticancer Research*.

[6] Kuan L. L., Tan L. T., Jepson S., Pollard C., Dennison A. R. (2020). A case of recurrent hepatic haemangioendothelioma. *Annals of the Royal College of Surgeons of England*.

[7] Zavras N., Dimopoulou A., Machairas N., Paspala A., Vaos G. (2020). Infantile hepatic hemangioma: current state of the art, controversies, and perspectives. *European Journal of Pediatrics*.

[8] Wahab M. A., Nakeeb A. E., Ali M. A. (2018). Surgical management of giant hepatic hemangioma: single center’s experience with 144 patients. *Journal of Gastrointestinal Surgery*.

[9] Iacobas I., Phung T. L., Adams D. M. (2018). Guidance document for hepatic hemangioma (infantile and congenital) evaluation and monitoring. *The Journal of Pediatrics*.

[10] Farhat W., Ammar H., Said M. A. (2021). Surgical management of giant hepatic hemangioma: a 10-year single center experience. *Annals of Medicine and Surgery*.

[11] Leon M., Chavez L., Surani S. (2020). Hepatic hemangioma: what internists need to know. *World Journal of Gastroenterology*.

[12] Zhang L., Chen X. J., Lee J. M., Lin S. S. (2018). Hepatic epithelioid hemangioendothelioma: challenges in the preoperative diagnosis. *The Kaohsiung Journal of Medical Sciences*.

[13] Hau H. M., Kloss A., Wiltberger G. (2017). The challenge of liver resection in benign solid liver tumors in modern times - in which cases should surgery be done?. Die Herausforderung der Leberresektion bei soliden benignen Lebertumoren in der heutigen Zeit – wann kommt eine Operation in Frage?. *Zeitschrift für Gastroenterologie*.

[14] Xie Q. S., Chen Z. X., Zhao Y. J., Gu H., Geng X. P., Liu F. B. (2021). Outcomes of surgery for giant hepatic hemangioma. *BMC Surgery*.

